# Neural Network Model of Dynamic Prediction of Cross-Border E-Commerce Sales for Virtual Community Knowledge Sharing

**DOI:** 10.1155/2022/4286148

**Published:** 2022-08-21

**Authors:** Hui Guan

**Affiliations:** ^1^Foreign Language Department, Changzhi University, Changzhi, Shanxi 046000, China; ^2^GSB, Universiti Kebangsaan Malaysia, 43600 UKM, Bangi, Selangor, Malaysia

## Abstract

The current popular one with forecasting method simply studies for prediction, and insufficient consideration is given to the prediction of the evolution of product sales applied to Internet platforms. To improve the forecast effect and to realize the usage of the forecasting in line with “Internet+” surroundings, the product sales controllable correlation mining, personalized forecasting ways of counting, improve counting, and other corresponding algorithms, a “Internet + foreign trade” concept based on the controllable correlation comes up with the model of mobile prediction. The result can show that the sample has the opening features and dynamics of “Internet+” to prerealize the dynamic, intelligent, and quantitative qualitative prediction of export product sales based on the controllable correlation big data of cross-border e-commerce in the “Internet + foreign trade” environment. The comprehensive prediction effect of this model is obviously better than that of traditional models and has strong evolution and high practical value. This thesis has the benefits for promoting the technological development of cross-border e-commerce and making us cross the cross-border e-commerce industry.

## 1. Introduction

In the “Internet + foreign trade” environment, activities will be more complicated, sales forecast of export products is affected by demand, customs, material flows, risks, and other factors, but the core of “Internet + foreign trade” is big data for prediction advantages, which make it relatively easy to predict the sales of export products [1]. The accurate, safe, and efficient sales forecasting model of export products driven by “foreign trade” based on controllable correlation has become a hot topic that has attracted much attention [2].

The global, decentralized, and virtual characteristics of e-commerce have counter-effected and promoted the applications [2]. The development of network technology and a wave of enterprise transformation and can bring about changes in society, which will change the mode of business activities, the way people used to spend, the government's office behavior, the production mode and operation mode of the enterprise, and generate new online financial models [3].

The transformation of traditional enterprises to e-commerce websites will be embodiment relationship for the market. For many enterprises, especially most of them with product sales as the main source of income, the network means an inexhaustible gold mine, and through the transformation to e-commerce websites, it is the most effective and direct mining method for traditional enterprises to mine this gold mine [4]. For e-commerce enterprises, the e-commerce market, as a branch of economics, can bring opportunities for rapid development for enterprises, and also make enterprises face associated challenges. On the one hand, the domestic or worldwide market competition has entered a white-hot stage, and enterprises must collect and use information to improve their business processing to adapt to the rapid changes in the business environment and improve the efficiency and quality of enterprises [5]. The development of computer networks and communication technology makes these applications possible, and e-commerce can employ means to organically coordinate the logistics, capital flow, and information flow in business activities, accelerate the process of business activities, for service quality and reducing transaction costs [6] as shown in Figure 1.

On the other hand, the transaction cost of the Internet is low, customers can choose freely between suppliers, and at the same time, it will lead to the transformation of the era of “information deficiency” to the era of “information democracy,” significantly reducing the degree of information asymmetry between economic entities, and even preventing toward a perfectly competitive market, bringing fierce price competition and meager profit space for enterprises [7]. Therefore, in the Internet era, the competition strategy and market initiative are no longer completely determined by enterprises, and at present, the training of enterprise talents and network infrastructure in China cannot fully meet the requirements, so the difficulty of enterprise profitability has become too much [8].

Although there are still difficulties in e-commerce, the Internet has brought the inherent characteristics of openness, low-cost, high-efficiency, and borderlessness to e-commerce, making e-commerce have the value of transcending as a new form of trade [9]. In the future, it is the entire society and even every business activity in the world [10].

The United States, Britain, France, Japan, and other developed countries have developed network popularity, social integrity system, and convenient logistics and transportation system, so that online electronic commerce has entered all levels of social life, and has achieved a certain degree of success [11]. Nowadays, with the popularization, many firms involved in this field have also built their own e-commerce system platform, the development potential is huge, but how to make good use of e-commerce platforms, improve the level of business is a value problem worth thinking about [12]. For small- and medium-sized e-commerce applications, the current level of technology application is low, and the integrity problem between merchants and customers has long plagued the development and growth of business, and in China will be in its infancy [13].

Within the last 30 years, domestic ones have ushered in a period of rapid development, and information and enterprise development have become directly equivalent factors [14]. The information technolgy became the core means of influencing the business of enterprises. and in the information age, it has become a profit expansion point. The continuous penetration of online business, changing the distribution business model and transforming to online business will help the development and growth of enterprises [15].

The dynamic prediction volume driven by “Internet + foreign trade” based on controllable correlation is proposed, which fully integrates the openness and extensibility of “Internet+,” so the application experiment is carried out [16]. It shows that the sales are based on cross-border e-commerce controllable correlation big data in the study [17].

## 2. State of the Art

Activities in the environment are more complex, and the sales forecast of export products is affected by various factors such as demand, tariffs, logistics, risks, but the core of the “Internet + foreign trade” business is big data with forecasting advantages, which make it relatively easy to predict the sales of export products. Therefore, the design of an accurate, safe, and efficient export product sales forecasting model based on cross-controllable correlation big data driven by “Internet + foreign trade” has become a hot topic that has attracted much attention. At present, KULKARNI excavates massive e-commerce data in third-party platforms based on big data classification methods, correlation grouping rules, online clustering methods, Internet big data matching principles, semantic analysis, and behavior analysis methods and establishes a product demand return prediction model based on big data classification methods, correlation grouping rules, online clustering methods, and Internet big data matching principles, semantic analysis, and behavior analysis methods. The literature HE Z Z used the historical sales data of cross-border e-commerce to establish a product sales forecast model; ATTIA uses quantitative and qualitative analysis methods based on historical data, prevalence, and new production customer value proposes a predictive model based on big data. The above research has a reference role, but due to the short time of the “Internet+” strategy, the “Internet+” powerful big data online prediction has emerged, and the above research does not have a more in-depth and effective study on how to integrate it into the dynamic wisdom sales in “Internet + foreign trade” environment [18].

In order to promote the innovative research and application of Internet+, and so on, this paper designs a quantifiable, dynamic, and intelligent forecasting for product sales based on cross-border e-commerce controllable correlation big data driven by cross-border e-commerce from the perspectives as shown in Figure 2.

## 3. Methodology

### 3.1. Definition of Controllable Correlation Sales Data

**Define 1 .**

Controllable correlation.

Controllable correlation refers to the nature of the controllable correlation between multiple phenomena that affect the results of a study [19]. The algorithm is as follows: suppose that *u* and *v* are two types of products, and the domain *I* = *I* ⋃ *I* is the quantitative space of “net + foreign trade,” as a set of phenomena. The data source vector *D* = (Iuv, Iuv, Iuv) in space; *I* = {I1, I2,…, In} is a collection of object items; Ui and vi ∈ I are a quantitative representation of the qualitative concepts uI and VI trust constraints. The *m* × *n*-order matrix *R* is the rating matrix for basic users. The certainty of *u* and *vμ* (*u*) and *μ* (*v*) ∈ [0, 1] are random numbers with a tendency to stabilize. A given target user a and its scoring vector A *μ* : *I* ⟶ [0, *n*], *u* ∈ *I*, *u* ⟶ *μ* (*u*). For i ∈ I, suppose that the attribute trust between the quantitative trust constraints *u* and *v* is S (ui, vi), and the largest *n* basic data of S (ui, vi) are combined. Enter two object messages to m1 and m2 for nonfalse public keys, and if the return value of m1 ∧ m2 is false, the controllable correlation between *m* and *m* is invalid. If the return value is nontrue, there is a controllable association between *m* and *m* [20].

**Define 2 .**

Controllable Correlation Sales Big Data.

Controllable correlation sales big data refer to big data that satisfy the above algorithm, and its algorithm is as follows: assuming that the score of big data item set of product *u* and target product *v* is I = {u|*i* ∈ N } and I = {v If I ≤ I, that is, for i ∈ I, all i ∈ I are established, and quantitative values *u*, v ∈ I is a random realization of the qualitative concept. Then all the scoring big data items of product *v* have been evaluated by product *u*, so *v* recommends controllable associations to *u.* If I > I, that is, for i ∈ I, both i ∈ I are valid, and the *μ*: I ⟶ [0, 1], with *u* ∈ I, *u* ⟶ *μ* (u), all the scoring big data items of product *u* have been producted, so the big data of product *v* must be controlled with *u* as shown in Figure 3.

### 3.2. The Sales Volume of Cross-Border E-Commerce Export Products Can Be Controlled and Correlated

Big data mining of export products in line with environmental platform (this platform is one, centralized in the National Internet Center) are mining policies, product types, total product demand of customers, trading groups, customer purchase psychology, payment, quotations, tariffs, inventory, logistics, orders, contracts, and commodity quality risks, returns or exchange rates, counterfeit and shoddy products, false publicity and other data. It is necessary to explore the key factors affecting the sales forecast of export products and the controllable correlation of big data. The mining model is shown in Figure 4.

The specific one

Step 1: design such online based on prediction behavior, conduct online estimation, and classification of big data of controllable correlation indicators affecting prediction, and determine the application of big data mining methods [21], but the blur phenomenon of data is not clearly characterized, and it is not integrated into Internet thinking, and the online classification function of Internet big data cannot be realized.

Hypothesis: on the basis of the Sections 3.1, 3.2 and 3.3 algorithm, given the data mining domain *C* and its nonempty subset

(1) $$\begin{array}{c} A,\left(C,A\right)=\left\{\left(C_{i},A_{i}\right)|i\in N_{+}\right\}. \end{array}$$

Defined as a set of confidence measures,

(2) $$\begin{array}{c} S=\left\{S_{i}=\left(S_{i1},S_{i2},S_{i3}\right)|i\in N_{+}\right\}. \end{array}$$

Equation 2 represents a collection of documents and logs on third-party platforms in the “Internet” environment {SAMi |i ∈ N} and SAB = {SABi|i ∈ *N*+} represent sets of data obfuscation and phenomena, respectively. The mapping function can be *F*1 = (FSi ⟶ FCi). If ∃*C*_*i*_ ∈ *C*∧(*C*_*i*_, *A*_*i*_)∧(*S*_*i*1_, *S*_*i*2_, *S*_*i*3_)∧*SAM*∧*SAB* ≠ False, the online classification and estimation method based on predicted behavior can be expressed using the function CF(*i*) as shown in equation (3):

(3) $$\begin{array}{c} CF\left(i\right)=\frac{A\left(1,n\right)\cdot \left|S_{i}\right|\cdot \left|FS_{i}\right|\cdot I_{uv}\cdot \mu \left(v_{i}\right)\cdot \sum_{i=1}^{n}SAM_{i}}{\left(I_{uv},I_{u},I_{v}\right)\cdot \mu \left(u_{i}\right)\cdot \left|C_{i}\right|\cdot \left|FC_{i}\right|\cdot \left|A_{i}\right|\cdot \sum_{i=1}^{n}SAB_{i}}. \end{array}$$

CF of ambiguity and some into different (*C*_*i*_, *A*_*i*_) phenomena. This is more characterized than the method before the improvement of the ambiguity.

Step 2: design such correlation and look for correlation between these correlations and organize. Correlation grouping rule is only the preliminary correlation of the data, and the correlation accuracy is low, so it needs to be improved and correlation is proposed.

For basis of the above equation, these are the possibility space and the measurement. Si is constrained by *t*_*i*_ in A set, and *ξ* is a fuzzy variable defined on K1. The expected value of the correlation is *ω*0. Meet such mapping “G:*K*1+K2 ⟶ K1, the constraint time of K2 represents a best search one degree that is denoted as *e*(*S*_*i*_, *S*_*j*_)=*b* − ∑_*x*=*i*_^*j*^*E*(*x*), and then the improved correlation rule available is the function as shown in (4) and represents

(4) $$\begin{array}{c} CV\left(S_{i},S_{j}\right)=\frac{\sum_{i=1}^{n}\sum_{j=1}^{m}e\left(S_{i},S_{j}\right)\cdot \xi \cdot \left(\left|CF\left(i\right)-K1\right|\right)}{\omega_{0}\cdot \prod_{i=1}^{n}\left(K2\cdot t_{i}\cdot T_{i}\cdot J_{i}\right)}. \end{array}$$

The role of the improved formula (2) is to accurately realize the correlation regularity between the big data product.

Step 3: design the similarity of the classified controllable correlation big data as large as possible, and then the data blocks are divided. In practical applications, K-means mean clustering is widely used in large sample datasets in distribution sets. Its algorithmic process is first, *k* samples are randomly selected as the starting center point; then, the samples other than the center point are placed in the cluster where the highest center point of similarity is located, and then the mean sample coordinates in the current cluster are established as the new center point; and then, according to the new center point, the loop continues to iterate until the category to which all samples belong no longer changes. In the online clustering method, however, the data blocks divided by the method are obviously crossed. Since this method holds the function of associative, this paper combines. Based on the definition of (2), it is assumed that the recommended weights of the predictor subject and object are *ω*1 and *ω*2, respectively. Clustering recommended sets are TJ = {tj1, tj2,…, tjn }, associated with the expected value of the description,

(5) $$\begin{array}{c} Q_{x}\left(tj_{i},tj_{j}\right)=TS\left(SAM_{ii},SAB_{i}\right)\cdot e\left(S_{i},S_{j}\right). \end{array}$$

Entropy value

(6) $$\begin{array}{c} Q_{n}\left(tj,tj\right)=\frac{TS\left(SAM_{ii},SAB_{i}\right)}{e\left(S_{i},S_{j}\right)}. \end{array}$$

Super-entropy value,

(7) $$\begin{array}{c} Q_{x}\left(tj_{i},tj_{j}\right)=TS\left(SAM_{ii},SAB_{i}\right)\cdot e\left(S_{i},S_{j}\right). \end{array}$$

Then improved online k-Means dynamic representation of the function shown in clustering and description method availability:

(8) $$\begin{array}{c} CVV\left(S_{i},S_{j}\right)=\frac{Qx\left(tj_{i},tj_{j}\right)\cdot \sum_{i=1}^{m}\sum_{j=1}^{n}\left(tj_{i}\cdot tj_{j}\cdot \left|\omega_{i}\cdot TJ\right|\right)}{Qn\left(tj_{i},tj_{j}\right)\cdot Qe\left(tj_{i},tj_{j}\right)\cdot CV\left(S_{i},S_{j}\right)}. \end{array}$$

The role of the improved (3) is that it can divide the similarity of the “Internet + foreign trade” cross-border e-commerce product sales data block as effectively as possible. Step 4 uses the Internet big data matching principles, semantic analysis, and behavior analysis methods proposed in the literature to retain the high signs of controllable correlation sales big data for the reasonable matching of major users, imports the key controllable correlation big data that affect the prediction through online or offline methods, integrates it into the Internet big data warehouse, cross-border e-commerce platform management background, and external application to integrate the key factors, and better solves the problem of the confusion of subject object attributes and the semantic control matrix reflecting the mapping between the domains of the prediction behavior.

### 3.3. Personalized Forecasting Mechanisms

According to the model shown in Figure 4, the following personalized prediction mechanism is constructed.

#### 3.3.1. Ways

Through the way, the accurate prediction of incremental dynamic evolution integration is realized, where it is as combinations of *M*_1_=*ω*_*i*_*CER*_*n*_^2^

#### 3.3.2. “Random Distribution-Association” Prediction Mechanism

However, for systems with stochastic model uncertainty and random external perturbations, distributed model predictions, the control method is still in the early stage of research, and there are still many key and difficult problems that have not been effectively solved. For example, how to coordinate the control behavior of each subsystem to ensure that the coupling constraints are satisfied and reduce the conservatism of constraint processing? How to use uncertainty information to design local, controllers that can ensure iterative feasibility and stability of the entire system, while reducing the amount of online computation. How to use the internal relationship between the overall control goal and the control quantity of each subsystem to achieve the overall optimization and coordination of the global system. Through machine learning, randomly distributed product sales data are correlated for prediction, where the random distribution factor attribute can represent tuple *Q* = (the mathematical combination of Bn − 1 and Bn), *B*_*n*_^2^ the combined number *M*2 = CERn^2^.

In order to achieve quantitative and qualitative personalized predictions, these two mechanisms need to be expressed mathematically. Its key data for new products are insufficient in terms of random distribution, correlation, evolution, and similarity assessment, so based on the definition and formula of controllable correlation big data in Section 1.1, the C&M-CVPDSS is improved.

Suppose that the reference sample libraries of personalized machine learning and neural networks are mint = {CER (C1C1), CER (C2 C2),…, CER (Ci). Cj)}, a random distribution, correlation, evolution problem set composed of market demand, trading market operation, transaction content integration problem set is AAT = {AAi |i ∈ *N*+}, data allocation function is *G* (Ci, C j) = (CER (CiCj)/*n*, m) tuple, then the it can be used as follows, respectively The mathematical function is shown to express:

(9) $$\begin{array}{c} DT=\frac{\sum_{i=1}^{n}\sum_{j=1}^{m}\left(\left|CER\left(C_{i},C_{j}\right)\right|\cdot \left|B_{j}\right|/G\left(C_{i},C_{j}\right)\right)}{Q\cdot B_{n}^{2}\cdot AA_{i}\cdot CVV\left(S_{i},S_{j}\right)}\\ DTT=\frac{\sum_{i=1}^{n}\sum_{j=1}^{m}\left(\left|AA_{i}\cdot CVV\left(S_{i},S_{j}\right)\right|\cdot G\left(C_{i},C_{j}\right)|/B_{j}\right)}{DT\;\cdot Q\cdot B_{n}^{2}\cdot CER\left(C_{i},C_{j}\right)}. \end{array}$$

Among them DT represents the transformation of automatic implementation indicators for concrete mechanisms; it represents automatic implementation of pattern, and associated indicators. The above formula automatically implements from abstract random distribution, correlation, to concrete mechanisms as well as pattern transformations.

### 3.4. Intelligent Prediction Algorithm for DPMES

DPME has become an important part of many classifiers, segmentation, human pose, and behavioral classification. DPME can be seen as an extension of HOG, and the general idea is consistent with HOG. The gradient direction histogram was computed first, and then the gradient model of the object was trained with SVM.

The DPMES dynamic predictive model is designed to identify problems with an organization. The results obtained from the analysis are used to guide operations personnel and managers to resolve any issues in the organization.

Step 1: press the CF(i) solution, according to the prediction direction, when the CF(i) value range is not an empty set, then the “Internet + foreign trade” environment can be controlled correlation export product sales big data source planning design and integration strategy as shown in the formula:

(10) $$\begin{array}{c} \left(C_{i},A_{j}\right):\left\{\left(C,A\right)\right\}\overset{CF\left(i\right)}{↔}FC_{i}:\left\{FC_{i}|i\in N_{+}\right\}. \end{array}$$

The influencing factors of controllable correlation prediction are extracted by using the formula, and the online one.

Step 2: Design a dynamic prediction wisdom integration strategy to dynamically add or delete prediction components. Calculate the definition range of the fuzzy variable by formula, extract the maximum value of DTT DTT, select several prediction components that meet the value range of [DTT, DT]. The integration policy can be expressed using the constraint coefficient *λ* shown in equation (11):

(11) $$\begin{array}{c} \lambda =\frac{\left(C_{i},A_{i}\right)}{FS_{i}:FC_{i}}. \end{array}$$

Step 3: Follow the above equation, extract all *ξ* in K1 and K2 that satisfy the threshold *ω*0 arbitrarily belonging to (C, A), looking for the best search time Ti. Discover this and based on the product ones, the correlation export product sales data are designed, and its function is shown in the above equation, that is, the membership degree *M* (Si, Sj, Tj) of CVV (S, S (tj, tj) is calculated:

(12) $$\begin{array}{c} M\left(S_{i},S_{j}\right)=CVV\left(S_{i},S_{j}\right)\cdot \lambda \cdot DT\;\cdot DTT. \end{array}$$

Step 4: divides the prediction behavior class BT and similarity between the *μ* (*x*) and *μ* (*y*) reaches the maximum value, and several target prediction behaviors with different scoring characteristics are classified into the subset of behaviors with different memberships in the same filter recommendation.

Step 5: designs the dynamic optimization prediction methods such as for most critical algorithms in this paper. The literature uses them to solve the problem of dynamic optimization and does not solve the distributed and centralized optimization calculation problems well. Each node dynamically selects the next cluster node according to all its neighbor nodes as shown in Figure 5 and Figure 6.

For this reason, the clusters, segments, and orphans are, in order

(13) $$\begin{array}{c} \left\{\begin{array}{c} HQ=\frac{{\left(CV{\left(S_{i},S_{j}\right)}^{T_{i}}\right)}^{-1/4}{\left(DT^{T_{i}}\right)}^{-1/2}{\left(CF{\left(i\right)}^{T_{i}}\right)}^{-1/3}}{M\left(S_{i},S_{j}\right)}\\ HF={\left(FS_{i}^{T_{i}}\right)}^{-1/3}{\left(CVV{\left(S_{i},S_{j}\right)}^{T_{i}}\right)}^{-1/2}{\left(DTT^{T_{i}}\right)}^{-1/4}\\ HG=CVV{\left(S_{i},S_{j}\right)}^{\lambda /2}CV{\left(S_{i},S_{j}\right)}^{\lambda }{\left(DTT^{\lambda }\right)}^{-1/3} \end{array}\right). \end{array}$$

Step 6: sets the (*C*_*i*_, *C*_*j*_)_max_ and (*C*_*i*_, *C*_*j*_)_min_ as maximum and minimum values of Ci Cj, respectively. Repeat steps 1 to 5 to fix the code characteristic C C of C in the threshold range [*ω*_*i*_, *ω*_*j*_], judgment (*C*_*i*_, *C*_*j*_)_max_ > *ω*_*i*_∧(*C*_*i*_, *C*_*j*_)_min_ < *ω*_*j*_

Step 7: Design the parallel synthesis prediction function formula shown in the equation:

## 4. Result Analysis and Discussion

### 4.1. DPMES Dynamic Prediction Model Construction

The model is designed to identify problems with the organization. The results obtained from the analysis are used to guide operations personnel and managers to resolve any issues in the organization. Using the above personalized prediction mechanism and intelligent prediction algorithm, the DPMES dynamic prediction model is constructed by using the decision tree, as shown in Figure 7.

The build path is as follows.

Firstly, according to step 1 of the intelligent prediction algorithm, the prediction target is determined and the data sample range for modeling is selected, and several factors with prediction characteristics and capabilities are screened and filtered.

Secondly, as for the random distributions, dynamically add or delete prediction components by using A. Integrate key factors, prepare, estimate, clean, nonlinear transformations, and validate data as shown in Table 1.

Then, according to the algorithm step 4, the collaborative filter recommendation is implemented, and the subset of prediction behavior is divided.

Third, according to the above formula, centralize the real-time tracking of controllable correlation big data streams; synthesize misalignment and alignment of the Internet big data search index, select the key data with the largest search index as the benchmark index, build a model, do online reallocation, give parallel big data weights and related coefficients, centralize qualitative prediction of which potential customers are most likely to become consumers and traders, and conduct significant tests on possible transaction clues. Distribute quantitative forecast of sales volume in the next cycle and real-time prediction of future sales structure trend of export products.

Finally, there is the model evaluation and application. Error analysis is performed on the prediction results of each forecasting method, and if the average error of the method on the prediction results of previous periods is greater when the method is synthesized, the more the method should have less influence on the comprehensive prediction results when the comprehensive forecasting is synthesized. The decision tree is further divided into leaf nodes according to the weights and related coefficients filtered out by the screening, and the comprehensive forecast value of sales volume can be obtained after the model is stabilized, and the optimization of inventory policy path is realized accordingly, and the model application is realized.

According to Figures 4 and 7, the front-end uses java (or C#/C+) and the back-end uses open source PHP and SQL Server to build a dynamic prediction system.

### 4.2. Experimental Data Collection

Data selection requires a good understanding of the business goals in order to model the goals. There are three types of data that can be used for modeling: demographics, behavior, and psychology. Preparing the data into the correct format for analysis is a very critical part. The model needs to be trained with previous data, and for this reason, the data may need to be cleaned. Variables should be well defined, and multiple datasets can be combined. The data used in this article are from January 2015 to July 2016 Alibaba AliExpress platform *v* China, the National Bureau of Statistics fixed product sales indicator statistics platform, and Zhejiang Cross-border e-commerce Public Service Platform and has 10,000 fixed data on leather shoes, machinery, electrical appliances, and other manufacturing export products within these three platforms, as well as some actual dynamic data outside the platform. According to the big data mining model in Section 1.2, the keyword mining tool is used to describe keywords from the two dimensions. The data analysis is shown in Table 2.

### 4.3. Comparative Analysis of Experimental Results

Experiment 1 uses more than 10,000 fixed data to verify the rationality of the improvement method, the personalized prediction mechanism based on the improved method, and the intelligent prediction algorithm. The process is as follows:

(1) Verify such product, *E*(*x*) = *b* is constrained by CF(*i*), membership is calculated, key data are randomly distributed, associated, evolution, integration of indexation and similarity evaluation, and verification of validity.
(2) Verifiable distributed quantification.
Such verification indicators and the feature point error (the difference between the controllable correlation characteristics of export product sales), the mismatch rate (the rate of correlation export product sales), and the mean square of Internet search error of the calculation formula are as shown in Table 3. In order to better express the error relationship, add *o* linear parameter (b, b,…, bn) equation (15), respectively. The functions represent as shown in Table 3:
  (14) $$\begin{array}{c} TXX\left(x\right)=\frac{TCZ\left(S_{i}\right)\cdot \sqrt{TCL\left(S_{i}\right)\cdot M{\left(S_{i},S_{j}\right)}^{\lambda }}}{{\left(CPW{\left(v,u\right)}^{\omega 0}+TCX{\left(S_{i}\right)}^{2}\right)}^{T_{i}}}\\ ZJS\left(x\right)=\frac{TCZ{\left(S_{i}\right)}^{b_{n}}\cdot TCL{\left(S_{i}\right)}^{\omega 0}}{WPR{\left(v,u\right)}^{T_{i}}\cdot \int_{0}^{b_{n}}KXX\left(x\right)}\\ WCXS\left(x\right)=\frac{APW\left(v,u\right)\cdot TCZ{\left(S_{i}\right)}^{\omega }\cdot NQQ{\left(x\right)}^{b_{n}}}{WPR\left(v,u\right)\cdot CPW{\left(v,u\right)}^{T_{i}}\cdot \prod_{x=1}^{n}KXX\left(x\right)}\\ KKD\left(x\right)=\frac{WCXS\left(x\right)\cdot WPR\left(v,u\right)\cdot APW\left(v,u\right)}{NQQ{\left(x\right)}^{b_{n}}\cdot \sum_{x=1}^{n}\left(KXX\left(x\right)\cdot ZJS\left(x\right)\cdot CPW\left(v,u\right)\right)}. \end{array}$$

The analysis of the validation results is shown in Figure 8. It can be seen from Figure 8.

Experiment 2 is based on Experiment 1, and still uses the above 10,000 fixed data for 10,000 experiments, and the average value obtained by the experiment is used as the result data, and the performance of DPMES is compared with the model established in the literature and the C&M-CVPDS model” and the product identification failure prediction model.

Its formula is represented by the function shown in the formula in order:

(15) $$\begin{array}{c} KXX\left(x\right)=\frac{TCZ\left(S_{i}\right)\cdot \sqrt{TCL\left(S_{i}\right)\cdot M{\left(S_{i},S_{j}\right)}^{\lambda }}}{{\left(CPW{\left(v,u\right)}^{\omega 0}+TCX{\left(S_{i}\right)}^{2}\right)}^{T_{i}}}\\ NQQ\left(x\right)=\frac{TCZ{\left(S_{i}\right)}^{T_{i}}\times TCL\left(S_{i}\right)⊕M{\left(S_{i},S_{j}\right)}^{\lambda }}{APW{\left(v,u\right)}^{\omega 0}⊗TCX{\left(S_{i}\right)}^{b_{n}}}\\ ZJS\left(x\right)=\frac{TCZ{\left(S_{i}\right)}^{b_{n}}\cdot TCL{\left(S_{i}\right)}^{\omega 0}}{WPR{\left(v,u\right)}^{T_{i}}\cdot \int_{0}^{b_{n}}KXX\left(x\right)}\\ WCXS\left(x\right)=\frac{APW\left(v,u\right)\cdot TCZ{\left(S_{i}\right)}^{\omega }\cdot NQQ{\left(x\right)}^{b_{n}}}{WPR\left(v,u\right)\cdot CPW{\left(v,u\right)}^{T_{i}}\cdot \prod_{x=1}^{n}KXX\left(x\right)}\\ KKD\left(x\right)=\frac{WCXS\left(x\right)\cdot WPR\left(v,u\right)\cdot APW\left(v,u\right)}{NQQ{\left(x\right)}^{b_{n}}\cdot \sum_{x=1}^{n}\left(KXX\left(x\right)\cdot ZJS\left(x\right)\cdot CPW\left(v,u\right)\right)} \end{array}$$

The experimental results are shown in Table 4.

From Table 4, it can be found, that when the product sales are hot, the forecast of the incremental index is closer to the stable and accurate actual forecast value. Conversely, the year-on-year decrease in sales volume hovers around the risk line whether it is a product sales expectation forecast indicator or an actual forecast indicator for the overall forecast.

(1) The mean squared error of the out-of-sample prediction of the fixed indicator is
  (16) $$\begin{array}{c} MSE\left(S_{i}\right)=\frac{KXX\left(x\right)\cdot WCXS\left(x\right)\cdot TCL{\left(S_{i}\right)}^{T_{i}\cdot e}}{KKD\left(x\right)\cdot TCZ{\left(S_{i}\right)}^{\lambda }\cdot MAE} \end{array}$$
(2) Parallel comprehensive fluctuation prediction efficiency.

In line with fixed data of several actual dynamic samples in the previous period, the same formula is used for the forecast time period in parallel to it, and so on.

(17) $$\begin{array}{c} YWR\left(x\right)=\frac{WCXS\left(x\right)\;⊕\;CPW{\left(v,u\right)}^{\lambda \cdot e}\cdot APW{\left(v,u\right)}^{T_{i}}}{TCZ\left(S_{i}\right)⊗NQQ{\left(x\right)}^{\lambda \cdot e}\cdot YWR\left(x\right)}\\ ZXCD\left(x\right)=\frac{KXX\left(x\right)/CPW{\left(v,u\right)}^{\lambda \cdot T_{i}}\cdot APW{\left(v,u\right)}^{T_{i}}}{TCZ\left(S_{i}\right)⊗NQQ{\left(x\right)}^{\lambda \cdot e}\cdot YWR\left(x\right)}\\ KCYR\left(x\right)=\frac{YWR\left(x\right)\cdot \sum_{i=1}^{n}\left(TCX\left(S_{i}\right)\cdot TCL{\left(S_{i}\right)}^{\lambda \omega }\right)}{APW{\left(v,u\right)}^{T_{i}}\cdot TCZ\left(S_{i}\right)\times ZXC\;D{\left(x\right)}^{\lambda \cdot e}} \end{array}$$

The forecast results are shown in Table 5. As can be seen from Table 5, the forecast value of sales volume in each quarter shows an upward trend, while the forecast error ratio, confidence level, and inventory optimization efficiency are basically within the acceptable range. Based on the parallel comprehensive forecast results of each quarter, the cumulative growth rate of each quarter can be calculated.

## 5. Conclusion

The DPMES prediction algorithm and model are based on the online method prediction behavior, such as correlation rule function. The other functions are based on the personalized prediction mechanism, and the methods are scientific and reasonable, and they solve some theoretical and practical problems, and also fully integrate the openness, extensibility, online and dynamic evolution of big data and prediction advantages of Internet+, and realize the “Internet+” parameters such as wisdom, export product correlation for cross-border e-commerce in the driving environment and have reference value for efficient marketing and efficient inventory planning of foreign trade enterprises, deepening the mining of data and information generated in e-commerce. The source data of e-commerce often hides a certain coupling relationship; we can purposefully collect statistics on customer behavior, order list, customer browsing behavior data in e-commerce activities in the data warehouse, extract and standardize, which is conducive to further product intrinsic association analysis, customer browsing behavior clustering analysis, business component multianalysis and other in-depth data mining, which helps to expand product sales and enhance the competitiveness of enterprises.

However, in view of the “Internet+,” big data are highly complex technologies. The research in this article only applies the Internet+ and big data technology, although the actual process has also been innovated in these computer science and technology, but it is not easy to achieve, thereby reducing the performance of the system to a certain extent, so in the future. The authors of this article will continue to research on the Internet+, cross-border e-commerce, big data technology and fusion algorithms.

## Figures and Tables

**Figure 1:** Importance of each feature.

**Figure 2:** Data analysis process.

**Figure 3:** Prediction process based on data mining.

**Figure 4:** The export products in the environment.

**Figure 5:** The multiple linear regression method.

**Figure 6:** Data analysis process.

**Figure 7:** DPMES dynamic prediction model 3 algorithm model application examples.

**Figure 8:** Improves the algorithm validation results to visualize scatter plots.

**Table 1:** Lag feature variable and sales volume correlation coefficient.

	Lag one-phase correlation coefficient	Significance	Lag two-phase correlation coefficient	Significance	Lag three-phase correlation coefficient	Significance
Sales volume	0.412	0.000	0.241	0.000	0.120	0.000
Flow rate	0.470	0.000	0.304	0.000	0.193	0.000
Inventory	0.225	0.000	0.197	0.000	0.182	0.000
SKU number	0.231	0.000	0.226	0.000	0.221	0.000
Direct reduction amount	0.394	0.000	0.239	0.000	0.109	0.038
Full reduction amount	0.365	0.000	0.210	0.000	0.077	0.146
Coupon amount	0.338	0.000	0.392	0.000	0.185	0.000
Additional purchase number	0.290	0.000	0.194	0.000	0.179	0.000
Additional collection number	0.316	0.000	0.215	0.000	0.186	0.000

**Table 2:** Experimental data analysis.

Controllable relevance indicators (keywords)	Sales concern (range: 10–15)	Factor attention
Product categories	9.976670 to 10.012,350	Main sales product share
Total customer demand	13.557320 to 13.687010	Ratio of major audience groups, product demand
Customer buying psychology	13.642350 to 13.75200	Interests, purchasing power and behavior ratio
Product cycle	10.547280 to 10.580150	Manufacturing, sales cycle
Inventory	10.469230 to 10.89905	Purchasing quantity, backlog, inventory quantity, cost, replenishment, shipping quantity, inventory balance and transfer, storage location
Price	14.682140 to 14.692050	Cross-border payments, quotations, insurance, duties, costs, profits
Logistics	10.467822 to 10.884332	Warehousing, transportation and distribution, supply chain costs
Risks	14.973471 to 14.981810	Product quality and performance, return or exchange rate, credit rating

**Table 3:** Predictive evaluation on training set.

Regression model	Characteristics	Parameters	R2	RME	MAPE
Linear regression	All	—	0.8693	5090	0.0675
Linear regression	12345678	—	0.8615	5214	0.0692
Random forest	All	ntree = 300		3008	0.0320
Random forest 2	12345678	ntree = 700		3237	0.0372
Support vector regression, linear	All	Kernel = “linear,” cost = 10, gamma = 0.0001	0.8557	5344	0.0646
Support vector machine linear 2	12345678	Kernel = “linear,” cost = 10, gamma = 0.0001	0.8513	5428	0.0664
Support vector machine nonlinear	All	Kernel = “radial,” cost = 100, gamma = 0.001		4872	0.0594
Support vector machine nonlinear 2	12345678	Kernel = “radial”, cost = 100, gamma = 0.001		5054	0.0630
BP neural network nonlinear	All	Size 18, maxit = 1000, linout = *F*		298	0.0041
BP neural network, nonlinear 2	12345678	size40, maxit = 1000, linout = *F*		4026	0.0577

**Table 4:** Performance comparison of various models.

Algorithm example	Reliability measure	Uncertainty distinction	Best search time (s)	Error factor	Controllable correlation
Literature [2] model	19.0	13.1	12.2	7.0	—
Literature [2] model	18.1	12.5	12.7	7.1	—
Literature [3] model	18.7	13.4	13.0	6.8	10.2
Literature [4] model	19.1	12.7	12.7	6.2	11.5
C&M-CVPDSS model	22.1	15.8	14.8	6.0	12.0
Product marking failure prediction model	19.7	13.3	13.5	6.0	12.5
DPMES	22.0	15.1	15.0	5.5	14.0

**Table 5:** Is based on DPMES predictions.

Quarterly	Expected value	Actual value	Predicted value	Prediction error ratio (%)	Confidence (%)	Inventory optimization efficiency (%)
1	21090	20240	20117	1.006	92.60	89.45
2	22588	23468	23240	1.010	92.18	90.51
3	24668	24889	24951	0.998	90.99	90.42
4	25850	25901	26001	0.996	93.50	91.30

## Data Availability

The labeled dataset used to support the findings of this study are available from the author upon request.
